# Effect of Holistic Nursing Intervention Combined with Humanized Nursing Intervention on Activities of Daily Living and Limb Movement Ability of Elderly Patients with Cerebral Hemorrhage after Surgery

This article has been retracted.

**DOI:** 10.1155/2021/2480551

**Published:** 2021-10-22

**Authors:** Lan Zhang, Haiyan Du, Jie Song

**Affiliations:** ^1^Department of Thoracic Surgery, Jiaozhou Central Hospital of Qingdao, Qingdao 266300, Shandong Province, China; ^2^Health Service Centre, Qingdao Fifth People's Hospital, Qingdao 266001, Shandong Province, China; ^3^Second Department of Health Care, Weifang People's Hospital, Weifang 261041, Shandong Province, China

## Abstract

**Background:**

To improve the nursing status, activities of daily living (ADL), and limb movement ability of elderly patients with cerebral hemorrhage and to actively explore the comprehensive nursing mode that can meet the rehabilitation needs of patients.

**Methods:**

128 elderly patients with cerebral hemorrhage admitted to our department (2019.01–2021.01) were included in the study and randomly divided into the reference group and the study group according to the numeration table, with 64 cases in each group. The reference group received routine nursing, while the study group received holistic nursing combined with humanized nursing. Statistical methods were used to analyze the nursing effect of the two intervention models.

**Results:**

With better scores of the upper limb muscle strength, lower limb muscle strength, and total Fugl-Meyer Assessment (FMA) in both groups after nursing, the scores in the study group after nursing were higher than those in the reference group (*P* < 0.05). After nursing, the ADL scores of both groups were significantly improved and the score in the study group was better than that in the reference group (*P* < 0.05). After nursing, the degree of neurological deficit in both groups was significantly better than that before nursing and the degree in the reference group was more serious than that in the study group (*P* < 0.05). Compared with the reference group, the total infection rate in the study group was lower, while the nursing satisfaction was higher, with statistical significance (*P* < 0.05).

**Conclusion:**

The holistic nursing combined with humanized nursing has a remarkable effect on the postoperative intervention of elderly patients with cerebral hemorrhage. It can improve the limb movement function, enhance the ADL, reduce the degree of neurological deficit, improve the quality of life, and enhance the nursing satisfaction of patients after intervention, which is worthy of clinical popularization.

## 1. Introduction

Senile cerebral hemorrhage refers to the hemorrhage caused by nontraumatic vascular rupture in the brain parenchyma, which is related to cerebrovascular diseases [1–4]. In addition, long-term hypertension and diabetes may also cause cerebral amyloid angiopathy followed by hemorrhage. Cerebral hemorrhage is generally in large amount and spreads over a wide area. However, because of the brain atrophy in elderly people, senile cerebral hemorrhage generally does not endanger the life of patients but affects their limb movement function and activities of daily living (ADL). Therefore, effective nursing intervention should be combined with clinical treatment [5–8]. Basic nursing measures such as cleaning of respiratory tract, blood pressure control, and observation of sign changes are often implemented for such patients in clinical practice, which leaves unsatisfactory nursing effect and low nursing satisfaction. Humanized nursing is a nursing method developed on the basis of conventional nursing. This method is patient-centered, aiming at the disease and development of patients, personality characteristics, cognitive level, and service needs to develop humanized nursing programs to meet the humanized needs of patients and provide high-quality clinical nursing services. Relevant studies have suggested that the humanized nursing intervention during perioperative period of patients with cerebral hemorrhage can significantly improve their dysfunction in limb movement, swallowing, and cognition [9, 10]. Holistic nursing mode is the nursing mode with high clinical implementation rate at present. Its purpose is to provide the most comprehensive, systematic, and scientific nursing intervention according to patients' conditions and lay the foundation for patients' rapid recovery on the basis of meeting patients' basic needs for clinical nursing work. Holistic nursing intervention can improve patients' quality of life after intervention, but its effect on postoperative limb movement ability and ADL of patients has not been reported. Therefore, this study explored the effect of holistic nursing combined with humanized nursing on ADL and limb movement ability of elderly patients with cerebral hemorrhage after surgery, aiming to improve the nursing status and clinical nursing effect.

## 2. Materials and Methods

### 2.1. General Information

128 elderly patients with cerebral hemorrhage admitted to our department (2019.01–2021.01) were included in the study and randomly divided into the reference group and the study group according to the numeration table, with 64 cases in each group.

The general data of patients in the two groups were statistically analyzed (*P* > 0.05), indicating comparability (Table 1).

### 2.2. Inclusion Criteria

(1) All patients were diagnosed with cerebral hemorrhage by brain CT examination and met the clinical diagnostic criteria for cerebral hemorrhage in the *Chinese Guidelines for the Prevention and Treatment of Cerebrovascular Diseases*; (2) the patients were no less than 60 years old; (3) the patients had high compliance and complete medical records; (4) the patient has normal comprehension and language skills; and (5) patients were able to cooperate with the research. This study was approved by the hospital ethics committee, and the family members of the patients knew the study and signed the informed consent.

### 2.3. Exclusion Criteria

(1) The patients were complicated with severe organ and tissue lesions or malignant tumors, (2) the patients' vital signs were unstable, and (3) the patients were unable to participate in the study due to communication or mental disorders.

### 2.4. Methods

The reference group received routine nursing measures, including medication guidance, diet nursing, psychological intervention, and environmental nursing [11–13].

The study group received the holistic nursing combined with humanized nursing, and the holistic nursing combined with humanized nursing team was established. Each team was led by 1 head nurse and assisted by 3 nurses. All team members received professional training and took up their posts after passing the assessment. Personalized care plan was developed according to the individual situation of patients. The specific measures are as follows. (1) The nursing staff analyzed the disease in detail and imparted disease-related knowledge to the patients and their families, timely answered the patients' questions, made preoperative preparations, and informed the patients and their families of intraoperative and postoperative precautions to accelerate the changes in the behaviors and consciousness of patients. (2) The staff assisted patients to establish healthy behaviors, control their blood pressure and blood glucose levels, improve their compliance during surgery, alleviate the negative emotions through active communication, enhance confidence, and actively participate in the treatment [14–16]. (3) Health behavior plans were formulated according to the patients' condition to reduce risk factors. The staff actively communicated with patients' family members and cooperated with them to encourage the patients. The patients were instructed to take medicine following the doctor's advice and reduce bad behaviors. (4) After reasonable assessment of the patients' condition, rehabilitation training plans were developed, so that the patients could fully realize the importance and necessity of healthy behaviors and keep healthy behaviors, thus enhancing the rehabilitation effect after intervention. (5) The staff instructed the patients to keep scientific diet, strengthened postoperative follow-up, timely solved their difficulties, and enhanced social and family support to monitor their health behaviors, to ensure the continuity of health behavior and reduce the risk of bad behaviors.

### 2.5. Observation Indexes

#### 2.5.1. Limb Movement Function

The Fugl-Meyer Assessment (FMA) score was used to evaluate the upper and lower limb motor function of patients. The total score of FMA was 100 points, and the total score of upper and lower limbs was 66 and 34 points, respectively. A higher score represented stronger limb function.

#### 2.5.2. ADL

According to the Activities of Daily Living Scale, the scale included daily living ability, including bathing, eating, personal hygiene, dressing, urination control, toilet transfer, transfer of a chair and bed, flat walking, and walking up and down stairs, scoring 0–100 points. A higher score represented better ADL.

#### 2.5.3. Neurological Deficit Score

The neurological deficiency scale (NIHSS) developed by the National Institutes of Health (NIH) was adopted. The total score of NIHSS scale was 31 points, and there were 13 items. A higher score represented more serious neurological deficit.

#### 2.5.4. Infection

Various infections in both groups were recorded during nursing, and the infection rate was calculated for statistical analysis.

#### 2.5.5. Nursing Satisfaction

The self-made questionnaire in our hospital was used, with a total score of 100 points. The self-made questionnaire of our hospital included daily communication, health education, nursing operation ability, and nursing service attitude. The score was positively correlated with satisfaction.

### 2.6. Statistical Treatment

In this study, the data were processed by SPSS 20.0 software. The data included numeration data and measurement data, which are expressed as (*n* (%)) and ($\bar{x}$ ± *s*) and tested by the *χ*^2^ test and *t*-test. The difference was statistically significant when *P* < 0.05.

## 3. Results

### 3.1. Statistical Analysis of the Limb Motor Function in the Two Groups

With better scores of the upper limb muscle strength, lower limb muscle strength, and total FMA in both groups after nursing, the scores in the study group after nursing were higher than those in the reference group, with statistical significance (*P* < 0.05; Table 2).

### 3.2. Statistical Analysis of ADL in the Two Groups

After nursing, the ADL scores of both groups were significantly improved and the score in the study group was better that in the reference group, with statistical significance (*P* < 0.05; Table 3).

### 3.3. Statistical Analysis of Neurological Deficit Scores in the Two Groups

After nursing, the degree of neurological deficit in both groups was significantly better than that before nursing and the degree in the reference group was more serious than that in the study group, with statistical significance (*P* < 0.05; Table 4).

### 3.4. Statistical Analysis of the Infection in the Two Groups

The total infection rate in the study group was lower than that in the reference group, with statistical significance (*P* < 0.05; Table 5).

### 3.5. Statistical Analysis of Nursing Satisfaction in the Two Groups

The nursing satisfaction score in the reference group was significantly lower than that in the study group, with statistical significance (*P* < 0.05; Table 6).

## 4. Discussion

Cerebral hemorrhage results from a variety of causes, in which the most common one is hypertension combined with atherosclerosis. In addition, cerebral amyloid angiopathy, arteriovenous malformations, and various hematological diseases may also lead to cerebral hemorrhage [17–20]. Cerebral hemorrhage is a type of cerebrovascular disease with the highest fatality rate that reaches 30–40% in the acute stage. After surgical treatment, the patients' condition tends to be stable, often leaving different degrees of disability, such as language and sensory and motor function disorders. In order to fundamentally guarantee the prognosis of patients with cerebral hemorrhage, appropriate nursing modes are explored for them in the clinical medicine. In recent years, many scholars have affirmed the intervention effect of humanized nursing in postoperative nursing of elderly patients with cerebral hemorrhage because it can help them to actively improve the symptoms of respiratory system and endocrine system and provide a better rehabilitation environment for them [21–24]. On this basis, this study additionally adopted the holistic nursing mode in order to carry out a comprehensive management model for elderly patients with cerebral hemorrhage.

Benjamin's team enrolled 204 cancer patients into the study, receiving routine care in the reference group and holistic care intervention in the study group. The results of the study found that the patients in the study group had higher knowledge scores and had a better understanding of disease conditions and knowledge about signs and symptoms [25]. Garza-Hernandez's research showed that for surgical patients, nursing requires not only scientific, academic, and clinical nurses, but also humanitarian and moral agency. Through a survey of 150 surgical patients, the results found that 67% of the participants think human care is beneficial [26]. In this study, with better scores of the upper limb muscle strength, lower limb muscle strength, and total FMA in both groups after nursing, the scores in the study group after nursing were higher than those in the reference group. After nursing, the ADL scores of both groups were significantly improved and the score in the study group was better than that in the reference group. After nursing, the degree of neurological deficit in both groups was significantly better than that before nursing and the degree in the reference group was more serious than that in the study group. Compared with the reference group, the total infection rate in the study group was lower while the nursing satisfaction was higher, which was consistent with the research of Kneihsl et al. [27]. These results suggest that the holistic nursing combined with humanized nursing is an effective auxiliary means for the treatment of elderly patients with cerebral hemorrhage and can effectively improve the limb motor function and neurological dysfunction of patients. The reasons are analyzed as follows. (1) Health is fundamental to the survival of elderly patients with cerebral hemorrhage, which includes not only physical health but also many aspects such as psychology and spirit. The holistic nursing combined with humanized nursing effectively improves the balance of the body system through comprehensive management measures, creates a good rehabilitation environment, and promotes the establishment of good health management consciousness in patients. (2) The nursing model further implements the *Outline of Health Education and Health Promotion Work Plan*, actively optimizes the health resource allocation, effectively solves the problems and difficulties that may occur in cerebral hemorrhage disease, and helps patients develop scientific and healthy living and hygienic and psychological habits. (3) The holistic nursing and the humanized nursing have a synergistic effect, which can jointly improve the clinical manifestations of elderly patients with cerebral hemorrhage, promote their rapid rehabilitation, and reduce the incidence of complications, providing comprehensive nursing measures in line with the rehabilitation needs of patients.

In conclusion, the holistic nursing combined with humanized nursing has a remarkable effect on the postoperative intervention of elderly patients with cerebral hemorrhage. It can improve the limb movement function, enhance the ADL, reduce the degree of neurological deficit, improve the quality of life, and enhance the nursing satisfaction of patients after intervention, which is worthy of clinical popularization.

## Figures and Tables

**Table 1:** Statistical analysis of patients' general information (*n*, $\bar{x}$ ± *s*).

Analysis indexes	Reference group (*n* = 64)	Study group (*n* = 64)	*χ* ^2^/*t*	*P*
Age range (years)	60–86	61–85		
Average age (years)	73.28 ± 8.15	72.89 ± 7.85	0.2757	0.7832
Body mass index (kg/m^2^)	22.54 ± 4.52	22.49 ± 4.60	0.0620	0.9506
Amount of bleeding (ml)	55.61 ± 9.72	55.54 ± 9.36	0.0415	0.9670
Preoperative Glasgow coma score (points)	8.18 ± 2.24	8.23 ± 2.21	0.1271	0.8991
Gender			0.1270	0.722
Male	35 (54.69%)	37 (57.81%)		
Female	29 (45.31%)	27 (42.19%)		
Underlying diseases			0.2976	0.585
Hypertension	41 (64.06%)	38 (59.38%)		
Diabetes	23 (35.94%)	26 (40.63%)		
Bleeding sites			0.1296	0.719
Basal ganglia	25 (39.06%)	27 (42.19%)		
Thalamus	16 (25.00%)	17 (26.56%)		
Cerebellum	10 (15.63%)	8 (12.50%)		
Cerebral ventricles	8 (12.50%)	8 (12.50%)		
Cerebral lobes	5 (7.81%)	4 (6.25%)		
Smoking (*n*)	33 (51.56%)	36 (56.25%)	0.2830	0.595
Drinking (*n*)	40 (62.50%)	42 (65.63%)	0.1357	0.713
Surgery types			0.1357	0.713
Craniotomy	40 (62.50%)	42 (65.63%)		
Minimally invasive surgery	24 (37.50%)	22 (34.38%)		
Education			0.1296	0.719
Junior high school and below	37 (57.81%)	39 (60.94%)		
Above junior high school	27 (42.19%)	25 (39.06%)		
Residence			0.4013	0.526
Urban area	48 (75.00%)	51 (79.69%)		
Rural area	16 (25.00%)	13 (20.31%)		

**Table 2:** Comparison of limb motor function ($\bar{x}$ ± *s*, points).

Indexes		Reference group (*n* = 64)	Study group (*n* = 64)	*t*	*P*
Scores of upper limb muscle strength	Before nursing	1.44 ± 0.39	1.47 ± 0.35	0.0214	0.9829
	After nursing	2.61 ± 0.42	3.45 ± 0.47	10.6613	≤0.001

Scores of lower limb muscle strength	Before nursing	1.88 ± 0.39	1.91 ± 0.42	0.4187	0.6761
	After nursing	3.01 ± 0.48	3.83 ± 0.56	8.8941	≤0.001

Total FMA scores	Before nursing	20.43 ± 2.35	20.36 ± 2.28	0.1710	0.8645
	After nursing	50.25 ± 7.44	62.81 ± 8.53	11.3801	≤0.001

**Table 3:** Comparison of ADL scores ($\bar{x}$ ± *s*, points).

Group	Before nursing	After nursing	*t*	*P*
Reference group (*n* = 64)	37.58 ± 10.17	55.24 ± 12.06	8.9555	≤0.001
Study group (*n* = 64)	38.11 ± 10.25	65.32 ± 12.46	13.4918	≤0.001
*t*	0.2936	4.6504		
*P*	0.7695	≤0.001		

**Table 4:** Comparison of NIHSS scores ($\bar{x}$ ± *s*, points).

Group	Before nursing	After nursing	*t*	*P*
Reference group (*n* = 64)	17.40 ± 1.55	13.04 ± 1.47	16.3279	≤0.001
Study group (*n* = 64)	17.35 ± 1.47	10.11 ± 1.09	31.6498	≤0.001
*t*	0.1872	12.8085		
*P*	0.8518	≤0.001		

**Table 5:** Comparison of occurrence of infection (*n* (%)).

Group	Pulmonary infection	Intracranial infection	Urinary system infection	Total infection rate
Reference group (*n* = 64)	5 (7.81)	2 (3.13)	4 (6.25)	11 (17.19)
Study group (*n* = 64)	1 (1.56)	0 (0.00)	1 (1.56)	2 (3.13)
*χ* ^2^				6.9351
*P*				0.008

**Table 6:** Comparison of nursing satisfaction ($\bar{x}$ ± *s*, points).

Group	Nursing satisfaction score
Reference group (*n* = 64)	78.51 ± 4.33
Study group (*n* = 64)	90.58 ± 4.22
*t*	15.9702
*P*	≤0.001

## Data Availability

The data are available from the corresponding author.

## References

[1] Starke R., McCarthy D., Chen C. (2020). Hemorrhage risk of cerebral dural arteriovenous fistulas following Gamma Knife radiosurgery in a multicenter international consortium. *Journal of Neurosurgery*.

[2] Cartmell S. C. D., Ball R. L., Kaimal R. (2018). Early cerebral vein after endovascular ischemic stroke treatment predicts symptomatic reperfusion hemorrhage. *Stroke: A Journal of Cerebral Circulation*.

[3] Ng P. P., Larson T. C., Nichols C. W., Murray M. M., Salzman K. L., Smith R. H. (2019). Intraprocedural predictors of post-stent retriever thrombectomy subarachnoid hemorrhage in middle cerebral artery stroke. *Journal of Neurointerventional Surgery*.

[4] Zhou X.-Y., Yu M., Cui H.-X. (2018). Correlation of the changes of blood brain barrier permeability with the activation of apoptosis, inflammatory response and stress response in rats with cerebral hemorrhage. *Journal of Hainan Medical University (English Version)*.

[5] Cheng Y. (2018). Value of individualized active rehabilitation training for neurological functional reconstruction in the convalescence of cerebral hemorrhage. *Journal of Hainan Medical University (English Version)*.

[6] Tang J., Jiang X.-G., Gong Y.-S. (2018). Effect of minimally invasive craniotomy combined with edaravone on cerebral oxygen metabolism, cerebrovascular function and oxidative stress in patients with acute cerebral hemorrhage. *Journal of Hainan Medical University (English Version)*.

[7] Zheng S.-S., Qian X.-Y., Li S.-Y., Zhao X. (2016). Interventional therapy of diabetes mellitus type 2 complicated with acute cerebral hemorrhage by using dexmedetomidine. *Journal of Acute Disease*.

[8] Gross B. A., Du R. (2017). Hemorrhage from cerebral cavernous malformations: a systematic pooled analysis. *Journal of Neurosurgery*.

[9] Riordan C. P., Orbach D. B., Smith E. R., Scott R. M. (2018). Acute fatal hemorrhage from previously undiagnosed cerebral arteriovenous malformations in children: a single-center experience. *Journal of Neurosurgery*.

[10] Luo F. (2017). Curative effect of surgery combined with nerve growth factor preparation treatment of acute cerebral hemorrhage. *Journal of Acute Disease*.

[11] Wang A. Y.-C., Hsieh P.-C., Chen C.-C. (2018). Effect of intracranial pressure control on improvement of cerebral perfusion after acute subarachnoid hemorrhage: a comparative angiography study based on temporal changes of intracranial pressure and systemic pressure. *World Neurosurgery*.

[12] Lai P. M. R., See A. P., Silva M. A. (2019). Noninfectious fever in aneurysmal subarachnoid hemorrhage: association with cerebral vasospasm and clinical outcome. *World Neurosurgery*.

[13] Kim B. J., Kwon S. U., Park J.-H. (2020). Cilostazol versus aspirin in ischemic stroke patients with high-risk cerebral hemorrhage. *Stroke*.

[14] Sakata H., Endo H., Fujimura M., Niizuma K., Tominaga T. (2020). Symptomatic cerebral hyperperfusion after cerebral vasospasm associated with aneurysmal subarachnoid hemorrhage. *World Neurosurgery*.

[15] Randell A., Daneshtalab N. (2016). Adjuvant-induced mono-arthritis potentiates cerebral hemorrhage in the spontaneously hypertensive rats. *Life Sciences*.

[16] Willeman T., Marlu R., Böhle H. (2018). Lethal cerebral hemorrhage after ticagrelor intoxication: a specific antidote is urgently needed. *Clinical Toxicology*.

[17] Morales-Fernandez A., Morales-Asencio J. M., Canca-Sanchez J. C., Moreno-Martin G., Vergara-Romero M., Group for Pain Management Hospital Costa del Sol Members (2016). Impact on quality of life of a nursing intervention programme for patients with chronic non‐cancer pain: an open, randomized controlled parallel study protocol. *Journal of Advanced Nursing*.

[18] Padykula B. M. (2017). RN-BS students’ reports of their self-care and health-promotion practices in a holistic nursing course. *Journal of Holistic Nursing*.

[19] Lyndon H., Latour J. M., Marsden J., Campbell S., Stevens K., Kent B. (2019). The holistic assessment and care planning in partnership intervention study (HAPPI): a protocol for a feasibility, cluster randomized controlled trial. *Journal of Advanced Nursing*.

[20] Robertz A.-C., Rudolfsson G. (2016). Tactile massage as a nursing intervention in child and adolescent psychiatry: nurses’ experiences. *Journal of Psychiatric and Mental Health Nursing*.

[21] Elaine S., Pandyasamta P. (2020). Spiritually sensitive intervention to mitigate depressive symptoms among hospitalized children affected with congenital heart diseases: insights for holistic pediatric nursing. *Journal of Holistic Nursing*.

[22] Högberg K. M., Sandman L., Nyström M., Stockelberg D., Broström A. (2018). Caring through web-based communication: a qualitative evaluation of a nursing intervention to create holistic well-being among patients with hematological disease. *Journal of Holistic Nursing: Official Journal of the American Holistic Nurses’ Association*.

[23] Chen J.-Q., Wang G.-S., Zhou Y.-J. (2021). The mechanism of the combination of radix paeoniae rubra-cortex moutan in treating cerebral hemorrhage based on network pharmacology. *Journal of Hainan Medical University (English Version)*.

[24] Li D., Chen Q.-X., Zou W. (2020). Acupuncture promotes functional recovery after cerebral hemorrhage by upregulating neurotrophic factor expression. *Study on Nerve Regeneration in China (English Version)*.

[25] Benjamin L. S. (2020). Holistic nursing upon the knowledge on care during myelosuppression among cancer patients. *Asian Pacific Journal of Cancer Prevention*.

[26] Garza-Hernández R., Melendez-Méndez C., Castillo-Martínez G., González-Salinas F., Fang-Huerta M. d. l. Á., Hidalgo H. C. (2020). Surgical patients’ perception about behaviors of humanized nursing care. *Hispanic Health Care International*.

[27] Kneihsl M., Niederkorn K., Deutschmann H. (2018). Increased middle cerebral artery mean blood flow velocity index after stroke thrombectomy indicates increased risk for intracranial hemorrhage. *Journal of Neurointerventional Surgery*.

